RETRACTED

# Short- and Long-Term Influences of Benzodiazepine and Z-Drug Use in Patients with Bipolar Disorder Combined Sleep Disturbance during Affective Period: A Nine-Month Follow-Up Analysis

**DOI:** 10.1155/2022/6799898

**Published:** 2022-05-30

**Authors:** Yiming Chen, Fan Wang, Lvchun Cui, Haijing Huang, Shuqi Kong, Nuoshi Qian, Mengke Zhang, Dongbin Lyu, Meiti Wang, Xiaohua Liu, Lan Cao, Yiru Fang, Wu Hong

**Affiliations:** ^1^Shanghai Mental Health Center, Shanghai Jiao Tong University School of Medicine, Shanghai, China; ^2^Shanghai Key Laboratory of Psychotic Disorders, Shanghai, China; ^3^CAS Center for Excellence in Brain Science and Intelligence Technology, Shanghai, China

## Abstract

**Background:**

Sleep disturbances and benzodiazepine (BZD)/Z-drug use are common in patients with bipolar disorder (BD).

**Objective:**

To investigate the short- and long-term effects of BZD/Z-drug use during acute affective episode.

**Methods:**

Participants diagnosed with BD as well as sleep disturbance chose BZDs/Z-drugs or not at will. Manic and depressive symptoms were assessed by Mental Disorders Questionnaire (MDQ) and Quick Inventory of Depressive Symptoms (QIDS) as self-reporting surveys. The participants were assessed by trained evaluators at baseline and months 1, 3, 6, and 9.

**Results:**

61 patients with BD combined sleep disturbances were studied. At baseline, patients who used BZDs/Z-drugs had more amount of mood stabilizers (*p* = 0.038), other psychotropic medications (*p* = 0.040), and more risk of suicide attempt (*p* = 0.019). The BZD/Z-drug group had a significantly higher QIDS reductive ratio as compared with the no BZD/Z-drug group at month 1; no significant differences in the variability of MDQ, QIDS reductive ratio, or recurrence rate were found between these two groups at baseline, month 1, month 3, month 6, or month 9.

**Conclusions:**

During acute affective episode, patients with BD combined sleep disturbance who took BZDs/Z-drugs tended to use more amount of mood stabilizers. Polytherapy of BZDs/Z-drugs or other psychiatric drugs could increase suicide attempt during an acute affective episode. BZD/Z-drug use, however, had a significant effect on helping depressive symptoms alleviate during affective period.

## 1. Introduction

Bipolar disorder (BD) is a recrudescent mood disorder with episodes of depression and mania [1, 2]. It is often associated with significant impairment in cognitive functioning, circadian rhythm abnormalities, decreased quality of life, and reduced life expectancy [3, 4]. One of the central features in BD is sleep disturbance [1, 5], with anxiety disorder being among the most highly prevalent comorbidities. Unfortunately, comorbid anxiety disorders are linked to more affective relapses, increased suicidality, sleep disturbances, and increased barriers to effective treatment [6]. Benzodiazepines (BZDs) are taken by 25%-90% of patients with BD [7] to manage anxiety and insomnia [8], despite their potential serious adverse effects, such as cravings, withdrawal symptoms upon discontinuation, and increased falls, especially in long-term use [9]. There is also evidence that BZDs have direct depressogenic effects, which may be particularly harmful to individuals with BD [10]. These side effects may be the reason why patients with sleep disturbance are unwilling to comply with the administration of these drugs. On the other hand, because of their proven efficacy, reduced side effects, and lesser concerns about addiction, non-BZD receptor agonists, such as zaleplon, zolpidem, and zopiclone (so-called Z-drugs), have become the most commonly prescribed hypnotic agents approved to treat sleep-onset and sleep-maintenance insomnia [11]. However, the spectrum of adverse effects is reportedly similar between Z-drugs and BZDs [12]. Several studies have indicated that patients of BD who used BZDs regularly showed higher levels of treatment resistance to mood stabilizers and have a greater risk of both manic and depressive relapses independent of the effects of comorbid anxiety and insomnia [13, 14]. Furthermore, BZD use might be associated with greater risk for recurrence of an affective episode among patients with bipolar I and II disorders [15]. The other factors related to BZD/Z-drug use especially during affective episodes, such as suicidality and psychotic symptoms, are currently unknown.

RETRACTED

The aim of this study was to investigate the effect of BZD/Z-drug use in patients with BD combined sleep disturbance during acute affective period and long-term effect of variability of depressive or manic symptoms during consolidation period.

## 2. Materials and Methods

### 2.1. Study Design and Patient Recruitment

Patients who met the inclusion and exclusion criteria were consecutively recruited and interviewed from May 1, 2013, to May 1, 2014, in Shanghai Mental Health Center. The study was approved by the Ethics Committee at Shanghai Mental Health Center. All participants were interviewed at the baseline and months 1, 3, 6, and 9.

### 2.2. Inclusion and Exclusion Criteria

The inclusion criteria were as follows: (1) over 18 years old; (2) meeting the Diagnostic and Statistical Manual of Mental Disorders, fourth edition, text-revision (DSM-VI TR) [16] criteria for BD, type I or type II, and sleep disturbance; (3) having emotional events from twelve months to three months before the first interview; and (4) signing the informed consent. Patients were excluded if they (1) were unable to complete the self-assessments and (2) had participated in any intervention study one or more years prior.

RETRACTED

### 2.3. Data Collection

All participants received psychiatric screening interviews from trained psychiatrists. In the interview session, the clinicians interviewed the participants in an interview room using the doctor-rating assessment questionnaire. All clinicians were well-trained for this project to ensure assessment consistency. Participants completed the Mental Disorders Questionnaire (MDQ) and Quick Inventory of Depressive Symptoms (QIDS) as self-reporting surveys in the same interview room with a clinician present, should any questions arise.

The doctor-rating assessment questionnaire also collected the following data:

- Identification number, age, and sex of the subject
- Admission and discharge dates of previous hospital visits
- Onset and termination dates of each affective episode
- Dates of initiation and cessation of all psychiatric drugs and dosage of each drug during each affective episode
- Other conditions present during an affective episode, such as suicide attempt and/or psychotic symptoms

### 2.4. Statistical Analyses

The subjects were grouped into the cohort using BZDs/Z-drugs and those not. Descriptive statistics were used to summarize patient characteristics. Variability of MDQ and QIDS reductive ratio in months 1, 3, 6, and 9 were compared using the Mann–Whitney *U* test. The associations between each predictor variable and the initiation of BZD/Z-drug administration were investigated using logistic regression modelling. Associations were estimated as odds ratios (ORs) with 95% confidence intervals (CIs). The effect of each variable was adjusted for the effects of all other variables in a full model, from which variables with a strong correlation to one or several other variables were removed. All statistical analyses were performed in statistical software IBM SPSS Statistics for Windows, version 22.0 (IBM Corp., Armonk, N.Y., USA). Statistical tests were two-tailed, and significance was set at *p* < 0.05.

## 3. Results

### 3.1. Differences in Demographic and Clinical Characteristics between the BZD/Z-Drug Group and the No BZD/Z-Drug Group

Seventy patients who met the inclusion and exclusion criteria were recruited into this study, with a median age of 30 years. Among them, 61 patients (85.7%) had sleep disturbances, including difficulty falling asleep, midnight awakening, early-morning awakening, and hypersomnia. Patients with sleep disturbances were selected for analysis. 33 (54.1%) patients took BZDs/Z-drugs for treatment while 28 (45.9%) did not. The number of completed follow-up cases was as follows: 1-month (*n* = 61, 100%), 3- month (*n* = 61, 100%), 6-month (*n* = 60, 98.4%), and 9-month (*n* = 60, 98.4%) (Figure 1). The clinical characteristics of the 61 patients with sleep disturbance are presented in Table 1. The two groups showed no significant differences in age, sex, number of each type of emotional episode, duration of current episode, family history of mental illness, history of somatic diseases, combined mental illnesses, or previously diagnosed mental illnesses.

RETRACTED

Among BZD/Z-drug users, 29 patients took one BZDs/Z-drugs and 4 patients took two BZDs/Z-drugs. The median duration of using BZDs/Z-drugs was 30 days. Based on their classification under the European Monitoring Centre for Drugs and Drug Addiction [17], the BZDs were divided into either short- or long-acting drugs. Of the patients who received a prescription for a BZD or Z-drug, 13 (28.3%) had received a long-acting substance, whereas 30 (65.2%) had a short-acting substance, with the remaining 3 (6.5%) having had Z-drugs. The application of BZDs/Z-drugs in males and females is shown in Table 2. No significant differences were found between the male and female groups.

### 3.2. Association between Other Psychotropic Drugs and BZD/Z-Drug Use at Baseline

All of the study participants took at least one type of psychotropic drug other than BZDs/Z-drugs at baseline, for a total of 316 psychotropic drug prescriptions. Most participants were on multiple drugs, with a median of four different drugs per patient (interquartile range: 3-6 drugs). Notably, 31 participants were on five or more regular psychotropic drugs. However, among the 61 participants with sleep disturbance, 28 did not choose BZDs/Z-drugs. Between the BZD/Z-drug group and the no BZD/Z-drug group, we found a significant difference in the amount of mood stabilizer use at baseline (*p* = 0.038) but not in month 1 (*p* = 0.269), month 3 (*p* = 0.895), month 6 (*p* = 0.723), or month 9 (*p* = 0.741). The amounts of the other psychotropic drug types used at baseline did not show any significant difference between the two groups. These results are presented in Table 3.

### 3.3. Association between Suicide Attempt and the Number of BZDs/Z-Drugs and Other Psychiatric Drugs

Among the variables considered for multiple logistic regression analysis, the number of BZDs/Z-drugs and other psychiatric drugs remained in the model as independent risk factors of suicide attempt at baseline. Patients who took more than one type of BZD/Z-drug were more likely to have a suicide attempt than those who took only one type (OR = 4.338, 95% CI: 1.068-17.623, *p* = 0.040). Similarly, patients who took more than one type of other psychiatric drugs were more likely to have a suicide attempt than those who only took one type (OR = 1.835, 95% CI: 1.105-3.047, *p* = 0.019) at baseline. However, with regard to the appearance of psychotic symptoms at baseline, age, sex, hospitalization status, type of affective episode, and number of psychiatric drugs, they did not have any significant effect.

RETRACTED

### 3.4. Variability of Manic and Depressive Symptoms with and without BZDs/Z-Drugs in Short and Long Terms

The reductive ratio of total MDQ score was not significantly different between the two groups in month 1 (*Z* = −0.872, *p* = 0.383), month 3 (*Z* = −0.940, *p* = 0.347), and month 6 (*Z* = −1.251, *p* = 0.211). The reductive ratio of total QIDS score was not significantly different between the two groups in month 3 (*Z* = −1.826, *p* = 0.068) and month 6 (*Z* = −0.729, *p* = 0.466), but was significantly in month 1 (*Z* = −2.049, *p* = 0.040) (Table 4).

During the nine-month follow-up, recurrence was observed among 31 participants. Of them, 5 were in the BZD/Z-drug group and 8 were in the no BZD/Z-drug group. Depressive episodes recurred among nine of them, whereas four had mixed episodes. However, the recurrence rate showed no significant difference between the BZD/Z-drug group and no BZD/Z-drug group (*χ*^2^ = 1.627, *p* = 0.227).

## 4. Discussion

In this study, during an affective episode, as well as at baseline, approximately 81.7% patients with BD had sleep complaints. Among them, approximately 45.9% who initiated treatment with BZDs or Z-drugs continued such treatment for a maximum of seven months. Notably, BZD/Z-drug use could reduce depressive symptoms during acute affective period. However, polytherapy with BZDs/Z-drugs or other psychiatric drugs already exists and was found to be a strong predictor for suicide attempt during an affective episode. Furthermore, a significant difference in the amount of mood stabilizers used was discovered between the two bipolar cohorts in our study, with or without BZD/Z-drug use.

One result of this study was that among the 33 patients who initiated BZD or Z-drug treatment, 90.9% used clonazepam, which is among the most commonly abused drugs worldwide [18]. Although warnings about the highly addictive properties of clonazepam have emerged in recent years [19], one explanation for the high rate of long-term use could be that this drug still plays a role in the management of acute anxiety attacks if first-line treatment options, such as antidepressants, have failed or cannot be used for some reason. Anxiety disorder often requires a long treatment duration, illustrated by a lower-than-expected proportion of patients with comorbid anxiety disorder in our study. Although Z-drugs were initially perceived as having little or no abuse potential, more recent data show that Z-drugs are associated with considerable psychological and physiological dependence and abuse [20]. Among the BZD/Z-drug users, only one male used clonazepam continuously for more than six months, representing a yearly incidence of long-term BZD use of 3.6% among BZD/Z-drug users with BD. Hence, a certain level of vigilance is needed regardless of BZD/Z-drug prescription.

RETRACTED

On the other hand, while the BZD initiation rate was unaffected, the amount of mood stabilizers was significantly greater in the BZD/Z-drug group than in the no BZD/Z-drug group during the acute affective period. This may seem somewhat difficult to explain, given that the type of mood attack had been unrelated to BZD/Z-drug use. However, anxiety is a common symptom during depressive and mixed episodes and can be seen as an integral part of bipolar illness. Anxiety symptoms may also persist between affective episodes along with subsyndromal affective symptoms [21]. As anxiety is associated with a more severe illness course [22], these hard-to-treat symptoms might sometimes require choosing the lesser of two evils by, for instance, applying regimens of mood stabilizers and BZDs, despite their potentially harmful effects. Another explanation is the direct depressogenic effects of BZDs [10], which may be one cause of emotional instability. Based on these findings, the use of more mood stabilizers and even more antidepressants could be feasible.

Furthermore, we found that polytherapy with BZDs/Z-drugs increased the risk of suicide attempt among patients with BD during acute affective period. One previous study has presented a link between BZD treatment and past suicidal behavior in BD [23], although no distinction was made between short-term and long-term uses. In addition, anxiety is also associated with increased suicidality [22], as patients have anxious symptoms during an affective episode (such as depressive and mixed episodes) and experience a greater possibility of having these symptoms combined suicidal ideation, which then leads to the treatment of anxiety by using BZDs. Other retrospective studies, on the other hand, indicated that a history of self-harm also increased the risk for long-term BZD/Z-drug use [24, 25].

Unfortunately, our finding that BZD/Z-drug use was not a marker for a more severe course of illness is partly inconsistent with that of Perlis et al. [15]. This difference might due to our inclusion of Z-drugs, which led to the sole effect of BZDs not being observed.

RETRACTED

Despite the best efforts, a conclusive finding on the influences of BZD/Z-drug use for long term could not be provided, as BD is complex and variable. Although every aspect of the clinical features of BZD/Z-drug use were attempted to be covered during acute affective episode, the questionnaire did not provide a broad range of information in the strict sense. Another evident limitation of this study is that all of the questionnaires evaluating the aspects of depressive and manic severity are patient-reported. Hence, patient answers may not reflect the objective evaluations from clinicians and thus lead to some one-sided results. Moreover, due to their illness, some patients may not have answered the questions seriously, which may cause biases in our data. Fortunately, the clinicians who participated in this study were all well-trained to accurately record information to minimize the biases.

## 5. Conclusions

In this prospective study, the BZD/Z-drug use could effectively help alleviate depressive symptoms during acute affective period but had no significant effect on either recurrence rate, manic, depressive symptoms for long term. Polytherapy of BZDs/Z-drugs or other psychiatric drugs was predicted to increase suicide attempt during an acute affective episode. Also, BZD/Z-drug users appeared to take a greater amount of mood stabilizers than non-BZD/Z-drug users. Ultimately, the influence of BZD/Z-drugs use needs to be further explored among patients with BD combined sleep disturbance in both short and long terms.

## Figures and Tables

**Figure 1:** Study design flowchart.

**Table 1:** Demographic and clinical characters of patients at baseline.

	BZD/Z-drug group	No BZD/Z-drug group	*Z*/*t*/*χ*^2^	*p*
Sample size	33 (54.1%)	28 (45.9%)	/	/
Gender (male)	19 (67.9%)	17 (51.5%)	0.062	0.506
Age (median, interquartile range)	32 (21.5-45.5)	31 (24-38.5)	-0.043	0.965
Occupational status (employed/temporarily employed/unemployed)	15 (45.5%)/2 (6.1%)/16 (48.5%)	11 (39.3%)/1 (3.6%)/16 (57.1%)	0.543	0.762
Years of schooling (median, interquartile range)	12 (9-15)	12 (9-15)	-0.415	0.678
Residence (solitary/cohabiting)	1 (3.6%)/27 (96.4%)	0 (0.0%)/33 (100.0%)	1.198	0.459
Number of (hypo)manic episodes (%)	15 (68.2%)	7 (31.8%)	2.748	0.116
Number of depressive episodes (%)	16 (50.0%)	16 (50.0%)	0.455	0.609
Number of mixed episodes (%)	2 (28.6%)	5 (71.4%)	2.075	0.231
Episode duration (days) (interquartile range)	71.5 (48.5-127.5)	120 (60-170)	-1.655	0.098
Having family history of mental illness	1 (3.57%)	1 (3.03%)	0.014	0.711
Having history of somatic diseases	2 (7.14%)	3 (9.09%)	0.436	0.421
Combined anxiety disorder (%)	1 (3.57%)	1 (3.03%)	0.014	0.711
Combined substance abuse (%)	1 (3.57%)	2 (6.06%)	0.201	0.562
Combined eating disorder (%)	1 (3.57%)	1 (3.03%)	0.014	0.711
Previously diagnosed with PTSD (%)	0	1 (3.03%)	2.437	0.207
Previously diagnosed with periodic psychosis (%)	1 (3.57%)	0	0.863	0.541
Previously diagnosed with dissociative disorder (%)	0	1 (3.03%)	1.198	0.459
MDQ score	26.18 ± 2.82	26.75 ± 2.55	-0.826	0.412
QIDS score	11.94 ± 8.85	12.14 ± 7.29	-0.098	0.922
QIDS' score	8.36 ± 7.10	8.39 ± 5.85	-0.018	0.986

PTSD: posttraumatic stress disorder; MDQ: Mental Disorders Questionnaire; QIDS: Quick Inventory of Depressive Symptoms; QIDS': Quick Inventory of Depressive Symptoms, from questions 5 to question 16.

RETRACTED

**Table 2:** Treatment characteristics of BZD/Z-drugs.

	BZDs/Z-drugs	Number (%)	Male (%)	Female (%)	*χ* ^2^	*p*
Short-acting BZDs	Total number	13 (100.0%)	5 (38.5%)	8 (61.5%)	2.847	0.090
	Alprazolam	3 (23.1%)	0 (0.0%)	3 (23.1%)	4.810	0.057
	Lorazepam	9 (69.2%)	4 (30.8%)	5 (38.5%)	1.121	0.304
	Estazolam	1 (7.7%)	1 (7.7%)	0 (0.0%)	0.660	0.606

Long-acting BZDs	Clonazepam	30 (100.0%)	20 (66.7%)	10 (33.3%)	0.810	0.463

Z-drugs	Total number	3 (100.0%)	2 (66.7%)	1 (33.3%)	0.076	0.636
	Zolpidem	2 (66.7%)	1 (33.3%)	1 (33.3%)	0.096	0.637
	Zopiclone	1 (33.3%)	1 (33.3%)	0 (0.0%)	0.660	0.606

BZDs: benzodiazepines.

**Table 3:** Amounts of each psychotropic drug between two groups at baseline.

	BZD/Z-drug group	No BZD/Z-drug group	*Z*	*p*
Number (%)	33 (54.1%)	28 (45.9%)	/	/
Mean rank of mood stabilizers	25.98	35.96	-2.070	0.038^∗^
Mean rank of atypical antipsychotics	29.16	33.87	-0.713	0.476
Mean rank of SSRIs	32.66	31.57	-0.177	0.859
Mean rank of SNRIs	30.72	32.84	-0.198	0.843
Mean rank of NaSSAs	31.28	32.47	-0.507	0.612
Mean rank of other antidepressants	31.26	32.49	-0.444	0.657
Mean rank of typical antipsychotics	30.74	32.83	-0.673	0.501
Mean rank of other anxiolytics	30.00	33.32	-1.890	0.059

SSRIs: selective serotonin reuptake inhibitors; SNRIs: serotonin-norepinephrine reuptake inhibitors; NaSSAs: noradrenergic and specific serotonergic antidepressants. ^∗^*p* < 0.05.

**Table 4:** Variability of MDQ and QIDS reductive ratio between two groups.

		BZD/Z-drug group	No BZD/Z-drug group	*Z*	*p*
MDQ	Month 1	29.20	33.13	-0.872	0.383
	Month 3	29.06	33.29	-0.940	0.347
	Month 6	28.00	33.56	-1.251	0.211
	Month 9	28.64	32.78	-0.931	0.352

QIDS	Month 1	35.72	25.96	-2.049	0.040∗
	Month 3	34.74	26.59	-1.826	0.068
	Month 6	31.95	28.72	-0.729	0.466
	Month 9	31.36	29.44	-0.434	0.664

QIDS'	Month 1	33.53	28.02	-1.218	0.223
	Month 3	34.97	26.32	-1.949	0.051
	Month 6	29.00	32.33	-0.794	0.427
	Month 9	30.18	30.89	-0.211	0.833

MDQ: Mental Disorders Questionnaire; QIDS: Quick Inventory of Depressive Symptoms; QIDS': Quick Inventory of Depressive Symptoms, from questions 5 to question 16. ^∗^*p* < 0.05.

RETRACTED

## Data Availability

The data will not be shared or made publicly available.
